# Association of Low High-Density Lipoprotein Cholesterol Levels with Poor Outcomes in Hepatitis B-Associated Decompensated Cirrhosis Patients

**DOI:** 10.1155/2021/9927330

**Published:** 2021-07-27

**Authors:** Xia He, XiaoYun Liu, SongQing Peng, Zhong Han, Jianjiang Shen, Ming Cai

**Affiliations:** Department of Clinical Laboratory, Shengzhou People's Hospital, Shengzhou Branch of the First Affiliated Hospital of Zhejiang University, Shengzhou, Zhejiang Province, China 312400

## Abstract

**Background:**

Lipid levels become decreased in cirrhotic patients and are correlated with disease severity. In the present study, we investigated the impact of serum high-density lipoprotein cholesterol (HDL-C) on prognosis in patients with HBV-associated decompensated cirrhosis (HBV-DeCi).

**Methods:**

The medical records of 153 HBV-DeCi patients were analyzed. Patients were separated into survivors and nonsurvivors according to their 30-day survival. Univariate and multivariate analyses were performed to identify predictors of poor outcomes, and the performance of these predictors was evaluated by receiver operating characteristic (ROC) curve analysis.

**Results:**

The 30-day mortality in the cohort was 18.9%. HDL-C levels differed markedly between survivors and nonsurvivors. On multivariate analysis, Model for End-stage Liver Disease (MELD) score and HDL-C level were identified as independent risk factors for mortality in HBV-DeCi patients. In the ROC analyses, the prognostic accuracy for mortality was similar between HDL-C (area under ROC curve: 0.785) and MELD score (area under ROC curve: 0.853).

**Conclusions:**

Low HDL-C level had a significant correlation with mortality in HBV-DeCi patients and can be used as a simple marker for risk assessment and selection of therapeutic options.

## 1. Introduction

In China, hepatitis B virus (HBV) is the predominant cause of liver cirrhosis [1]. Decompensated cirrhosis (DeCi) is a major cause of mortality in HBV patients and can be accompanied by various complications [2]. Although several treatments are available, DeCi patients have a high mortality rate [2, 3]. Therefore, early assessment of disease severity and prognosis is crucial for the selection of appropriate treatment strategies, because effective treatment can reduce mortality in HBV-DeCi patients.

The liver plays important roles in several stages of lipid synthesis, transport, and metabolism. Abnormalities in serum lipid levels are common in patients with advanced liver disease [4], especially changes in serum high-density lipoprotein cholesterol (HDL-C). For example, HDL-C was shown to be a convenient independent risk factor for adverse outcomes in cirrhotic patients [5] and to be associated with disease severity [6, 7]. Furthermore, low HDL-C was demonstrated to be an accurate indicator of hepatic function and prognosis in noncholestatic cirrhotic patients [8]. Recently, Cheng et al. [9] identified HDL-C as an independent predictor for poor short-term outcomes in HBV-associated cirrhosis patients with gastrointestinal bleeding. In light of these findings, we investigated whether serum HDL-C can predict unfavorable short-term outcomes in HBV-DeCi patients.

## 2. Materials and Methods

### 2.1. Patients

A total of 206 patients diagnosed with HBV-DeCi were retrospectively recruited from February 2018 to June 2020 at the Department of Hepatology, Shengzhou People's Hospital. The study was approved by the Ethics Committee of the hospital. DeCi was diagnosed on the basis of histological findings, clinical, laboratory, imaging data, and presence of ascites, variceal bleeding, encephalopathy, or hepatorenal syndrome [10]. Among the 206 patients, patients with (a) concurrent infection with other hepatotropic viruses or HIV (*n* = 25), (b) alcoholic liver disease (*n* = 5), (c) hepatocellular carcinoma (*n* = 6), (d) autoimmune disease (*n* = 4), (e) cardiac disease (*n* = 5), (f) heart failure (*n* = 3), and (g) lack of complete medical records (*n* = 5) were excluded. Finally, 153 patients were enrolled.

### 2.2. Data Collection and Follow-Up

The following baseline demographic and clinical data were collected from the patients' medical records: age, sex, total protein, serum albumin, alanine aminotransferase, aspartate aminotransferase, total bilirubin, creatinine, HDL-C, blood urea nitrogen, platelet count, hemoglobin, and international normalized ratio (INR). Laboratory parameters were measured in all subjects using fasting venous blood samples. Liver function was assessed by the Model for End-stage Liver Disease (MELD) score as previously described [11]. All HBV-DeCi patients were followed up for 30 days, and the 30-day mortality rate was determined.

### 2.3. Statistical Analysis

Continuous values were expressed as median (interquartile range) and analyzed by the Mann–Whitney *U* test. Categorical values were expressed as number and analyzed by Fisher's exact test. Correlations between variables were examined by Spearman's analysis. Univariate and multivariate analyses were performed to evaluate the relationships between clinical variables and prognosis in HBV-DeCi patients. The area under the receiver operating curve (AUC) was calculated to determine the prognostic accuracy of the identified variables for mortality. All statistical analyses were performed using SPSS version 18.0 or MedCalc version 14.8.1 software. Values of *P* < 0.05 were considered statistically significant.

## 3. Results

### 3.1. Study Population

A total of 153 HBV-DeCi patients were included in this retrospective study. The main clinical events for hospitalization were ascites in 110 patients (71.9%), variceal bleeding in 33 patients (21.6%), encephalopathy in 3 patients (2.0%), and hepatorenal syndrome in 16 patients (10.5%). As shown in Figure 1, HDL-C level had a significant positive correlation with albumin level (*r* = 0.297, *P* < 0.001) and a significant negative correlation with MELD score (*r* = −0.505, *P* < 0.001).

A total of 29 (18.9%) patients died within 30 days after admission. We divided the patients into two groups based on whether or not they survived. As shown in Table 1, there were no significant differences in total protein, alanine aminotransferase, creatinine, hemoglobin, platelet count, age, or sex between the survivors and nonsurvivors. However, marked differences were observed between the survivors and nonsurvivors for serum albumin, MELD score, aspartate aminotransferase, total bilirubin, INR, blood urea nitrogen, and HDL-C level (all *P* < 0.05).

### 3.2. Low HDL-C as a Prognostic Indicator in HBV-DeCi Patients

Univariate analyses revealed that high MELD score, low serum albumin, and low HDL-C were associated with poor outcomes in HBV-DeCi patients. On multivariate regression analysis, MELD score and HDL-C remained associated with mortality (Table 2). The prognostic accuracies of HDL-C and MELD score for prediction of mortality according to ROC curves are shown in Figure 2. For prediction of mortality, baseline MELD score had a cutoff value of 15.2, with a sensitivity of 78.9% and a specificity of 83.9%, while HDL-C had a cutoff value of 0.53 mmol/L, with a sensitivity of 72.4% and a specificity of 76.6%. The AUCs for MELD score and HDL-C were 0.853 and 0.785, respectively. The power for predicting mortality was similar between the two indices (*Z* = 1.260, *P* = 0.208).

### 3.3. Clinical and Laboratory Findings Related to HDL-C Levels

The HBV-DeCi patients were stratified into two groups based on the cutoff value for baseline HDL-C (≤0.53 mmol/mL, *n* = 50 vs. >0.53 mmol/L, *n* = 103). Patients with HDL − C ≤ 0.53 mmol/L had lower serum albumin, higher MELD score, higher alanine aminotransferase, higher aspartate aminotransferase, higher total bilirubin, higher INR, and higher mortality (Table 3).

## 4. Discussion

In this study, we identified a correlation between HDL-C level and severity of HBV-DeCi. We also confirmed that serum HDL-C level was an independent risk factor for 30-day mortality in HBV-DeCi patients.

The MELD score is widely adopted to evaluate the severity of liver dysfunction and predict the prognosis of patients with liver disease and employs serum creatinine, serum bilirubin, and INR [11]. In the present study, we found that nonsurvivors had lower HDL-C levels than survivors. Moreover, decreased HDL-C was independently associated with 30-day mortality in HBV-DeCi patients, with a similar predictive power to the MELD score. Because HDL-C is a single laboratory parameter, it is more readily available and more inexpensive to assess than the MELD score. Notably, previous studies identified associations of several objective indicators obtained in routine examinations with adverse outcomes in cirrhotic patients, including serum cystatin C [12], total bilirubin [13], and serum C-reactive protein [14]. Our study complements these studies and indicates that HDL-C can also be used to predict prognosis in HBV-DeCi patients.

There are several possible explanations for the association between serum HDL-C and adverse outcomes in HBV-DeCi patients. First, malnutrition may play a role. Some studies have identified correlations between serum lipid levels and nutritional status. It is well known that low albumin is often associated with malnutrition. Previous studies demonstrated that low albumin was a common complication in cirrhotic patients that could lead to ascites or edema, and accounted for increased mortality [15, 16]. In the present study, serum albumin at admission was lower in nonsurvivors than in survivors and a positive correlation was found between HDL-C level and albumin level. Furthermore, albumin was identified as a risk factor for mortality in the univariate analyses. Bories and Campillo [17] previously confirmed that low HDL-C was increased and other parameters for liver function were improved after 1 month of nutritional supplementation. Therefore, we speculate that the predictive value of HDL-C could be partly attributable to the nutritional status of patients with HBV-DeCi. Second, considering that the liver is the main organ for cholesterol and apolipoprotein synthesis, hepatic function will directly affect these serum levels as well as the outcomes in patients with liver diseases. We found that HDL-C was negatively correlated with MELD score and that low HDL-C was correlated with high mortality, suggesting that low HDL-C may be a predictive factor for liver injury severity and progression in HBV-DeCi patients. The third and most important reason is that the development and progression of HBV-DeCi are associated with inflammatory responses. Numerous studies have indicated that systemic inflammation frequently occurs in patients with advanced cirrhosis and is associated with poor outcomes [18, 19]. Furthermore, investigators have clarified that HDL-C generally acts as an anti-inflammatory lipoprotein [20–22] and that HDL can bind and neutralize bacterial lipopolysaccharides to promote the excretion of these products [23, 24]. There is also accumulating evidence that inflammation markedly modifies the composition and function of HDL, generating dysfunctional or even proinflammatory forms of HDL [25–29]. For example, during acute conditions such as sepsis, increased levels of serum amyloid A and secretory phospholipase A2 may contribute to decreased HDL-C levels by replacing some structural and functional HDL components [28, 29]. Furthermore, Trieb et al. [30] observed that sera from cirrhotic patients had reduced levels of HDL-C and profoundly suppressed the activities of several enzymes involved in HDL maturation and metabolism [30]. Based on these findings, we hypothesize that HDL may lose its anti-inflammatory properties and the dysfunctional HDL may contribute to the poor outcomes in HBV-DeCi patients. However, HDL metabolism and modulation are far more complex than originally thought, and we believe that HDL-C can be helpful for predicting the prognosis of HBV-DeCi patients.

This study has some limitations. First, the retrospective study design may have led to a selection bias. Second, HDL-C was not monitored during the follow-up period. Finally, we were unable to examine other serum lipids, such as triglycerides, total cholesterol, and low-density lipoprotein, which may have been helpful in establishing the mechanism underlying the present findings. Further verification in a multicenter prospective study is warranted.

In conclusion, our study demonstrates that HDL-C is a robust predictor of survival in HBV-DeCi patients. The prognostic value of HDL-C as a simple and inexpensive parameter was similar to that of the MELD score. Our findings may lead to improved ability for monitoring of high-risk cirrhotic patients. However, our findings need to be validated by additional studies.

## Figures and Tables

**Figure 1:** Scatterplots illustrating the correlations of serum HDL-C with Meld score (*r* = −0.505, *P* < 0.001) and serum albumin (*r* = 0.297, *P* < 0.001) in HBV-DeCi patients.

**Figure 2:** Receive operating characteristic curves showing the prognostic performances of serum HDL-C and Meld score for prediction of poor outcomes in HBV-DeCi patients.

**Table 1:** Patient characteristics at baseline.

	All patients (*n* = 153)	Surviving patients (*n* = 124)	Nonsurviving patients (*n* = 29)	*P*
Gender (female/male)	30/123	22/102	8/21	0.346
Age (years)	53.0 (46.0-63.0)	53.0 (46.0-63.0)	55.0 (47.8-61.5)	0.952
Total protein (g/L)	61.5 (56.5-66.8)	61.7 (57.8-67.2)	59.4 (52.4-65.9)	0.098
Albumin (g/L)	30.6 (26.4-34.6)	31.4 (27.4-35.1)	28.9 (23.7-31.2)	0.011
Alanine aminotransferase (U/L)	29.0 (16.0-43.0)	28.0 (15.5-39.0)	38.0 (22.3-57.0)	0.102
Aspartate aminotransferase (U/L)	42.0 (27.8-71.0)	40.5 (27.0-63.5)	54.0 (31.8-97.5)	0.038
Serum creatinine (*μ*mol/L)	74.0 (61.0-87.0)	73.5 (61.0-84.0)	92.0 (61.8-124.0)	0.065
Total bilirubin (*μ*mol/L)	36.0 (17.8-83.3)	31.5 (16.0-59.0)	117.0 (64.8-212.5)	<0.001
Blood urea nitrogen (*μ*mol/L)	5.8 (4.3-7.7)	5.5 (4.2-7.4)	7.2 (5.8-12.9)	0.002
INR	1.34 (1.18-1.61)	1.30 (1.16-1.51)	1.67 (1.50-1.90)	<0.001
HDL-C (mmol/L)	0.73 (0.45-1.07)	0.82 (0.57-1.20)	0.40 (0.16-0.62)	<0.001
Platelet (×10^9^/L)	66.0 (40.8-120.3)	65.5 (39.5-113.0)	72.0 (59.3-159.3)	0.208
Hemoglobin (g/L)	101.0 (84.0-117.3)	103.5 (83.5-118.0)	94.0 (87.5-113.3)	0.407
MELD score	11.4 (6.8-16.8)	9.9 (6.0-13.7)	19.7 (15.4-22.5)	<0.001

Data are expressed as number or median (interquartile range). Abbreviations: INR: international normalized ratio; HDL-C: high-density lipoprotein cholesterol; MELD: Model for End-stage Liver Disease.

**Table 2:** Logistic regression analyses to identify risk factors associated with mortality in patients with HBV-associated decompensated liver cirrhosis.

	Univariate			Multivariate		
	Odds ratio	95% CI	*P*	Odds ratio	95% CI	*P*
Albumin (g/L)	0.912	0.845-0.984	0.014			
MELD score	1.289	1.170-1.420	<0.001	1.242	1.122-1.376	<0.001
HDL-C (mmol/L)	0.047	0.011-0.207	<0.001	0.184	0.038-0.893	0.036
Blood urea nitrogen (*μ*mol/L)	1.002	0.986-1018	0.843			
Aspartate aminotransferase (U/L)	1.004	1.000-1.008	0.083			

Abbreviations: CI: confidence interval; MELD: Model for End-stage Liver Disease; HDL-C: high-density lipoprotein cholesterol.

**Table 3:** Clinical data according to HDL-C levels.

	Low group (HDL − C ≤ 0.53 mmol/L, *n* = 50)	High group (HDL − C > 0.53 mmol/L, *n* = 103)	*P*
Gender (female/male)	13/37	17/86	0.242
Age (years)	56.0 (47.0-64.0)	52.0 (46.0-62.0)	0.452
Total protein (g/L)	62.2 (57.5-67.6)	61.2 (56.4-66.5)	0.341
Albumin (g/L)	29.1 (24.3-31.7)	32.1 (27.7-35.5)	0.004
Alanine aminotransferase (U/L)	38.0 (19.0-74.0)	27.0 (16.0-36.8)	0.007
Aspartate aminotransferase (U/L)	71.0 (33.0-113.0)	36.0 (26.8-52.3)	<0.001
Total bilirubin (*μ*mol/L)	97.5 (34.0-199.0)	26.0 (16.0-45.5)	<0.01
Blood urea nitrogen (*μ*mol/L)	5.7 (4.2-7.8)	5.9 (4.4-7.7)	0.590
INR	1.64 (1.30-1.89)	1.26 (1.14-1.48)	<0.01
Serum creatinine (*μ*mol/L)	70.5 (59.0-92.0)	76.0 (62.0-86.8)	0.288
Platelet (×10^9^/L)	80.0 (39.0-138.0)	65.0 (41.3-113.3)	0.510
MELD score	15.4 (11.3-21.1)	9.8 (5.7-12.9)	<0.001
Hemoglobin (g/L)	100.5 (86.0-114.0)	102.0 (83.3-118.8)	0.639
30-day mortality (yes/no)	21/29	8/95	<0.001

Data are expressed as number or median (interquartile range). Abbreviations: INR: international normalized ratio; MELD: Model for End-stage Liver Disease.

## Data Availability

The data are available upon reasonable request.

## Abbreviations

AUCs: Areas under the curve
CI: Confidence interval
DeCi: Decompensated cirrhosis
HBV: Hepatitis B virus
HDL-C: High-density lipoprotein cholesterol
INR: International normalized ratio
MELD score: Model for End-stage Liver Disease score
ROC: Receiver operating characteristic.
